This article has been retracted.

# Circular RNA mmu_circ_0001598 Contributes to IL-1*β*-Induced Osteoarthritis Progression by Regulating miR-127-3p

**DOI:** 10.1155/2021/2793379

**Published:** 2021-12-07

**Authors:** Xierenguli Apizi, Dilibaier Talifujiang, Aziguli Kasimu, Xue Zhang, Aibibula Yiming, Xin Ma, Qingshan Song, Dequan Wang

**Affiliations:** Department of Pain Treatment, People's Hospital of Xinjiang Uygur Autonomous Region, Xinjiang Uygur Autonomous Region, Urumqi 830001, China

## Abstract

Osteoarthritis (OA), a chronic disease characterized by articular cartilage degeneration, is a leading cause of disability and pain worldwide. Accumulating evidence indicates that circular RNAs (circRNAs) play a critical role in various diseases, but the function of circRNAs in OA remains largely unknown. In this study, we found that circ_0001598 was significantly upregulated in chondrocytes treated with IL-1*β* and in cartilage tissue from mice with severed anterior cruciate ligament surgery (ACLT) induced OA models. Interference with circ_0001598 in vitro restored IL-1*β*-induced chondrocyte proliferation and apoptosis. Silencing circ_0001598 significantly alleviated ACLT-induced OA in mice. Mechanistically, knockdown of circ_0001598 affected chondrocyte proliferation, apoptosis, and matrix degradation by regulating miR-127-3p. Taken together, our results demonstrate the fundamental role of circ_0001598 and provide new ideas for the prevention and treatment of osteoarthritis.

## 1. Introduction

Osteoarthritis (OA) is one of the degenerative joint diseases with high teratogenic and disability rates in the world, which is mainly characterized by chondrocyte apoptosis and joint matrix degradation [1]. The incidence of OA mainly occurs in middle-aged and elderly people, and the clinical incidence increases gradually with the increase of age [2, 3]. Currently, there are no effective disease-modifying therapies available for OA because of a limited understanding of its pathogenesis. Therefore, joint replacement is still the main treatment for patients with advanced osteoarthritis [4, 5]. Most people think that the occurrence and development of osteoarthritis are related to age, body weight, mechanical injury, and biological factors, and they may also be related to biomechanical disorders caused by pathological changes of articular cartilage in vivo [6]. The occurrence and development of OA involve the whole cartilage tissue (including the cartilage, synovium, and underlying bone), of which the pathological changes are most closely related to cartilage tissue, and damage to cartilage tissue is closely related to chondrocyte apoptosis [7–11]. Excessive apoptosis of chondrocytes is harmful to articular cartilage. The apoptosis of a large number of chondrocytes leads to the decrease of chondrocyte density, which not only leads to the destruction of the cartilage scaffold itself but also causes the degeneration of the cartilage due to insufficient secretion of the extracellular matrix [12, 13]. The extracellular matrix, composed of type 2 collagen and proteoglycans, not only provides tensile strength and elasticity for articular cartilage but also provides an external environment for chondrocytes to survive. Therefore, degradation of the extracellular matrix will lead to the change of mechanical properties of cartilage on the one hand and the loss of the survival environment of chondrocytes on the other hand, leading to apoptosis of chondrocytes [14]. The vicious cycle caused by the interaction of chondrocyte apoptosis and extracellular matrix degradation is one of the important reasons for the continuous development and aggravation of OA [15]. Although an increasing number of efforts have been devoted to unraveling the pathological process of osteoarthritis, its molecular mechanisms are still unclear. As a result, there is an unmet medical need to find novel drug targets to develop more effective therapeutics.

Circular RNAs (circRNAs) are a class of noncoding RNAs produced by dorsal splicing of precursor mRNAs and are widely expressed in mammals with highly conserved, stable, and tissue-specific patterns [16]. Because circRNAs are highly expressed, structurally stable, and possess a large number of miRNA binding sites, they may be a “biological sponge”' for enriching miRNAs [17]. CircRNAs rely on miRNAs to function and may play an important regulatory role in the onset and progression of a variety of diseases, including OA [18]. For example, Liu et al. found that 71 circRNAs were differentially expressed in osteoarthritis and normal chondrocytes [19]. Li et al. stated that circ_0136474 increased in OA cartilage tissue and could inhibit chondrocyte proliferation and promote apoptosis [20]. Shen et al. found that circSERPINE2 inhibits OA progression by targeting miR-1271-5p and ERG to regulate ECM metabolism in human chondrocytes [21]. hsa_circ_0005105 regulates NAMPT by inhibiting the transcriptional activity of miR-26a, resulting in accelerated degeneration of the extracellular matrix (ECM) in OA [22]. CircRNA.33186 directly binds and inhibits miR-127-5p to influence ECM catabolism and protect chondrocytes to reduce OA [23].

In the present study, we explored the role of circ_0001598 in the development of OA. We found that circ_0001598 was significantly upregulated in IL-1*β*-treated chondrocytes and cartilage tissue of ACLT-induced OA mouse models. Subsequent functional experiments showed that circ_0001598 significantly attenuated OA by binding miR-127-3p involved in chondrocyte proliferation, apoptosis, and matrix degradation. Taken together, we revealed the fundamental role of circ_0001598 to provide a potential drug target for OA treatment.

## 2. Materials and Methods

### 2.1. Animal Experiments

Eight-week-old mice were injected intraperitoneally with tamoxifen (Sigma, 100 *μ*g/g body weight) for 5 consecutive days. Anesthesia with isoflurane was followed by ACLT surgery of the right knee to establish an experimental OA model. Control mice were subjected to sham surgery, and mice were executed at 4 or 8 weeks after surgery. In treatment experiments, 4 weeks after ACLT surgery, mice received IA injections of lentivirus-incorporated si-circRNA to counter circ_0001598 or negative control lentivirus (1 × 10^9^ pfu in a total volume of 5 mL once a week) for 3 weeks. Mice were executed at week 3 and analyzed. All animal experiments were approved by the animal ethics committee and were performed according to the guidelines of this committee.

### 2.2. Primary Chondrocyte Isolation and Culture

First of all, newborn mice were immersed in alcohol after death, and articular cartilage of hind limbs was separated under aseptic conditions and put into a Petri dish filled with PBS solution. The cartilage tissue was cut into pieces and washed with PBS solution containing double antibodies 3 times in a 25 cm^2^ culture flask. Then, 0.25% trypsin, 10–15 times the volume of cartilage, was added for 1-2 hours before digestion was terminated. And 0.02% type II collagenase was added and digested at 37°C for 12 hours before adding DMEM/F12 (Gibco) culture medium. Finally, the filtrate was collected with a 200-mesh filter and centrifuged at 1500 r/min for 5 min in a culture consisting of DMEM/F12 (Gibco), 10% fetal bovine serum (Gibco, North America) and 1% penicillin-streptomycin (Gibco, USA) at 37°C in a 5% CO_2_ incubator.

### 2.3. siRNA Transfection

siRNA specifically targeting circ_0001598 and lentiviruses that expressed knockdown constructs of circ_0001598 and miRNA inhibitor were designed and constructed by Geneseed (Guangzhou, China). The sequences of siRNAs used were as follows:

- si‐scramble, GUGCGAGGGGGUUGUAAUC
- si‐RNA‐1, CTGCTTCAGCTCCTGCAGCTT
- si‐RNA‐2, GCCGTTTCTGCTTCAGCTCCT
- si-RNA-3,CCGTTTCTGCTTCAGCTCCTG

Chondrocytes were transfected with certain vectors using Lipofectamine 2000 (Invitrogen) in accordance with the manufacturer's instructions and then were used for further experiments.

### 2.4. qRT-PCR

TRIzol^®^ reagent (Invitrogen) was used to isolate total RNA from chondrocytes. To synthesize first-strand cDNA, a PrimeScript RT Reagent Kit (Takara) was used. Then, quantification of circRNA, mRNA, and GAPDH gene was performed using SYBR Premix Ex Taq (Takara Bio) in a real-time detection system (ABI one-step plus). Primer sequences were as follows: GAPDH, F 5′-TACCCCCAATGTGTCCGTC-3′, R 5′-GCCCAAGATGCCCTTCAGT-3′; circ_0001598, F 5′-TCCAGGGAATGCTGTGAAGAG-3′, R 5′-GAGAATCCTGCTGGTCTCCTG-3′; miR127-3p, 5′-AACAAGTCGGTTCGAGTCTGC-3′, R 5′-CAGTGCAGGGTCCGAGGT-3′; COL2A1, F 5′-ACCTTGGACGCCATGAAA-3′, R 5′-GTGGACAGTAGACGGAGGAA-′; MMP13, F 5′-GGAAGACCCTCTTCTTCTCT-3′, R 5′-TCATAGACAGCATCTA CTTTGTT-3′. The internal reference for the other genes was GAPDH, and we used the 2^–ΔΔCT^ method for the analysis of gene expression.

### 2.5. Western Blot

Total proteins were extracted from chondrocytes or cartilage tissues with RIPA lysis buffer (CWBIO, China), and the concentration was measured using the BCA protein assay (Beyotime, China). Then, proteins were electrophoresed on SDS-polyacrylamide gel and transferred to nitrocellulose membranes (Millipore, Carrigtwohill, Ireland). After blocking with nonfat milk, the membranes were incubated with a primary antibody overnight at 4°C, washed, and then incubated with a secondary antibody for 1 h each at room temperature. The antibodies used were anti-collagen II (dilution 1 : 5,000; Abcam, UK), anti-MMP-13 (dilution 1 : 3,000; Abcam, UK), GAPDH (dilution 1 : 1,000; Abcam, UK), and goat anti-rabbit secondary antibody (dilution 1 : 5,000; Abcam, UK). The results were quantified, and the images were processed using ImageJ software. GAPDH was used as an internal loading control.

### 2.6. CCK-8

CCK-8 assay was performed to measure the effect of circ_0001598 on chondrocyte proliferation. For the CCK-8 assay, cells were transfected with siRNA for 48 hours and then inoculated into 96-well plates at a density of 2,103 cells per well. Absorbance at 450 nm was measured using a SpectraMax 250 spectrophotometer. Each sample was repeated three times.

### 2.7. TUNEL

Chondrocytes were cultured in 24-well plates with 1 × 10^5^ cells in each well, and cell scorching was assessed by TUNEL analysis. After the indicated treatments, chondrocytes were fixed and permeabilized with 4% paraformaldehyde and 0.1% Triton X-100. Chondrocytes were incubated with the TUNEL reaction mixture for 1 hour at 37°C in the dark and stained with DAPI for 15 minutes. Confocal laser scanning microscopy (FV300, Olympus, Japan) was used to detect the fluorescence of the cells.

### 2.8. Statistical Analysis

Data are expressed as the mean ± SD, and statistical analysis was performed by one-way ANOVA for multiple comparisons or by Student's *t*-test. *p* < 0.05 (two-sided) was considered statistically significant for all of the statistical calculations. All statistical analyses were performed with GraphPad and SPPS.

## 3. Result

### 3.1. Circ_0001598 Is Raised in Cartilage Tissues of the OA Mouse and Chondrocytes Stimulated by IL-1*β*

Figure 1 analyzes the correlation between circ_0001598 and osteoarthritis. To investigate the potential role of circ_0001598 in OA, we examined the expression of circ_0001598 in IL-1*β*-induced chondrocytes by qRT-PCR. Circ_0001598 was found to be significantly upregulated in IL-1*β*-treated chondrocytes in a dose-dependent manner compared to controls (Figure 1(a)). To evaluate the expression of circ_0001598 in vivo, we used ACLT surgery to induce OA. Next, the expression of circ_0001598, matrix metalloproteinase 13 (MMP-13), and collagen (COL2A1) in OA cartilage tissues was detected by qRT-PCR, and it was found that compared to controls, circ_0001598 expression level was significantly higher in OA cartilage tissues compared with the control group, especially in the severe OA group (Figure 1(b)). Meanwhile, the expression level of MMP-13 in the degraded cartilage matrix in osteoarthritis cartilage tissue was increased, while the expression level of COL2A1, the main collagen component in the cartilage matrix, was downregulated (Figures 1(c) and 1(d)). Taken together, these data suggest that circ_0001598 may be involved in the progress of OA.

### 3.2. Effects of Circ_0001598 on Proliferation and Apoptosis in IL-1*β*-Treated Chondrocytes

To test the biological function of circ_0001598 in chondrocytes, we designed small interfering RNAs to knock down circ_0001598 and verified the knockdown efficiency of 3 independent siRNAs by qRT-PCR (Figure 2(a)). We selected siRNA3 for subsequent experiments because it was the most effective siRNA. To test whether circ_0001598 regulates chondrocyte proliferation, we transfected chondrocytes with siRNA3 and then treated them with 10 ng/ml 1L-1*β* for 24 h and detected cell proliferation using Cell Counting Kit-8 (CCK-8). We found that chondrocyte proliferation was significantly reduced after 1L-1*β* treatment, while circ_0001598 partially reversed its effect (Figure 2(b)). Next, we used TUNEL to analyze whether circ_0001598 affected chondrocyte apoptosis. It was observed that, in chondrocytes, IL-1*β* treatment induced apoptosis, while circ_0001598 silencing significantly reduced the percentage of chondrocyte apoptosis compared to the control (Figures 2(d) and 2(e)). The qRT-PCR and western blot results showed that the expression level of MMP-13 was significantly increased after IL-1*β* treatment, while the expression level of COL2A1 was downregulated. After knockdown of circ_0001598, the expression of MMP-13 was significantly decreased at the mRNA and protein levels, while the expression of COL2A1 was significantly increased compared to NC siRNA (Figures 2(c), 2(f), and 2(g)–2(i)). These data suggest that knockdown of circ_0001598 promotes chondrocyte proliferation, inhibits IL-1*β*-treated chondrocyte apoptosis, and protects against IL-1*β*-induced OA in vitro.

### 3.3. Silencing Circ_0001598 Alleviates ACLT-Induced Osteoarthritis In Vivo

To investigate the in vivo role of circ_0001598 in the pathogenesis of OA, we injected circ_0001598 and control siRNA weekly for 4 weeks using articular cavity lentivirus in ACLT-operated mice. qRT-PCR analysis was performed to verify the knockdown efficiency of circ_0001598 after lentivirus injection (Figure 3(a)). qRT-PCR and western blot showed that MMP-13 expression was increased, and COL2A1 expression was decreased in knee cartilage of mice with osteoarthritis, which was significantly alleviated by silencing circ_0001598 (Figures 3(b)–3(f)). Taken together, these data suggest that in vivo silencing of circ_0001598 attenuates ACLT-induced osteoarthritis in mice.

### 3.4. Circ_0001598 Exerts Chondrocyte Biological Functions by miR127-3p

Considering that circRNAs have been demonstrated to serve as a sponge of miRNAs, we predicted the potential target miRNAs interacting with circRNA on StarBase software (http://starbase.sysu.edu.cn/). We have found that circ_0001598 possesses multiple binding sites at the seed region of miR-127-3p (Figure 4(a)). We found that the expression level of miR-127-3p was significantly downregulated in IL-1*β*-treated chondrocytes in a dose-dependent manner (Figure 4(b)). Next, we cotransfected si-circ_0001598 and miR-127-3p inhibitor into chondrocytes and then treated the cells with 10 ng/ml of IL-1*β* for 24 h. CCK-8 and TUNEL showed that knockdown of circ_0001598 promoted chondrocyte proliferation and inhibited chondrocyte apoptosis, while the effect of circ_0001598 was reversed by silencing miR-127-3p (Figures 4(c)–4(e)). qRT-PCR and western blot analysis showed that reduced MMP-13 expression and elevated COL2A1 expression caused by circ_0001598 silencing were restored (Figures 4(f)–4(i)). In conclusion, these results suggest that circ_0001598 contributes to the pathogenesis of OA via miR-127-3p.

## 4. Conclusion

Recently, circRNAs have been shown to regulate gene expression by sponging miRNAs. Han et al. found that circRNA-MTO1 directly binds to miR-9 and inhibits miR-9 activity thereby regulating hepatocellular carcinoma progression [24]. Zheng et al. reported that circHIPK3 acts as a sponge for miR-124 to play a role as a cell growth regulator [18]. Huang et al. reported that circ_0001598 plays a key role in breast cancer progression and the regulation of trastuzumab resistance phenotypes through miR-1184/PD-L1 signaling [25]. However, the role of circ_0001598 in OA is still unknown. In the current study, we verified the interaction of circ_0001598 with miR-127-3p. circ_0001598 regulates IL-1*β*-induced cell proliferation and apoptosis through the modulation of miR-127-3p.

In summary, our study elucidates that circ_0001598 is elevated in mouse OA cartilage tissue and IL-1*β*-stimulated chondrocytes. In vitro knockdown of circ_0001598 promotes chondrocyte proliferation and inhibits chondrocyte apoptosis, and in vivo intra-articular injection of circ_0001598 lentivirus significantly attenuates ACLT-induced OA. Mechanistically, circ_0001598 reversed IL-1*β*-mediated cell proliferation and apoptosis via miR-127-3p. This may provide a new strategy and direction for the treatment of osteoarthritis with important implications.

## Figures and Tables

**Figure 1:** Expression analysis of circRNA.33186 in osteoarthritis. (a) qRT-PCR analysis of circ_0001598 expression in primary chondrocytes stimulated with 0, 5, 10, 50, or 100 ng/mL for 24 h. (b) qRT-PCR analysis of circ_0001598 expression in ACLT-induced OA cartilage tissues. (c) qRT-PCR analysis of MMP-13 expression in ACLT-induced OA cartilage tissues. (d) qRT-PCR analysis of COL2A1 expression in ACLT-induced OA cartilage tissues.

**Figure 2:** Effects of circ_0001598 on proliferation and apoptosis in IL-1*β*-induced chondrocytes. (a) Expression analyses of circ_0001598 knockdown efficiency by three different si-circRNAs in chondrocytes. (b) The effect of circ_0001598 on cell proliferation in vitro was determined by the CCK-8 assay. (c, f) Effects of circ_0001598 inhibition on COL2A1 and MMP-13 mRNA levels were determined by qRT-PCR. (d, e) The effect of circ_0001598 on cell apoptosis was measured by TUNEL. (g–i) Effects of circ_0001598 inhibition on COL2A1 and MMP-13 protein levels were determined by western blot and statistical analysis of western blots.

**Figure 3:** Silencing of circRNA_0001598 in vivo alleviates ACLT-induced OA. (a) qRT-PCR analysis of circ_0001598 expression in knee articular cartilage from OA mice in different groups after surgery (*n* = 8). (b, c) qRT-PCR analysis of COL2A1 and MMP-13 expressions in knee articular cartilage from OA mice in different groups. (d–f) Western blot analysis of COL2A1 and MMP-13 expressions in knee articular cartilage from OA mice in different groups and statistical analysis of western blots.

**Figure 4:** Circ_0001598 exerts chondrocyte biological functions by miR-127-3p. (a) Binding sites between circ_0001598 and miR-127-3p. (b) qRT-PCR analysis of miR127-3p expression in primary chondrocytes stimulated with 0, 5, 10, 50, or 100 ng/mL for 24 h. (c) The effect of circ_0001598 on cell proliferation in vitro was determined by the CCK-8 assay. (d, e) Cell apoptosis was measured by TUNEL. (f, g) qRT-PCR analysis of MMP-13 and COL2A1 expressions in different groups. (h, i) Western blot analysis of COL2A1 and MMP-13 expressions in different groups and statistical analysis of western blots.

## Data Availability

The simulation experiment data used to support the findings of this study are available from the corresponding author upon request.
